# Association between ERCC1 Gene Polymorphism (rs11615) and Colorectal Cancer Susceptibility: A Meta-Analysis of Medical Image Fusion and Safety Applications

**DOI:** 10.1155/2022/9988513

**Published:** 2022-10-14

**Authors:** Min Liu, Zhifeng Qiu, Qi Yang

**Affiliations:** ^1^Department of Reproductive Medicine, First Affiliated Hospital, School of Medicine, Shihezi University, Shihezi, Xinjiang, China; ^2^Genetic Laboratory, Maternal and Child Health Care Hospital of Baiyun District, Guangzhou, Guangdong 510010, China; ^3^Clinical Laboratory, First Affiliated Hospital, School of Medicine, Shihezi University, Shihezi, Xinjiang, China

## Abstract

Colorectal cancer (CRC) is a malignant tumor of the colorectal mucosa epithelial tissue transformed. The fusion of data for medical imaging has become a central issue in such biomedical applications as image-guided surgery and radiotherapy. Currently, CRC has been one of the most threatening tumors affecting people's health worldwide. The excision repair cross-complementation group 1 (ERCC1) is a key enzyme for nucleotide excision repair (NER). Emerging epidemiological studies have indicated that the presence of colorectal cancer (CRC) may be relevant to the ERCC1 rs11615 genetic polymorphism. However, the results of ERCC1 rs11615 on CRC in these studies are controversial. We searched PubMed, Web of Science, Embase, CNKI, and CBM databases for the effects of ERCC1 rs11615 variant on CRC development. There was no meta-analysis focused on the diagnosis of colorectal cancer with ERCC1 rs11615 variant. We creatively carried out a meta-analysis of nine case-control studies and used Stata (version 12.0) software to integrate the pooled odds ratios (ORs) corresponding to a 95% confidence interval (CI) of overall and subgroup analysis. Our results suggest that a significant correlation was observed between rs11615 and the susceptibility of CRC OR 95% CI = 1.13 (1.04-1.23) under an allele genetic model and OR 95% CI = 1.14 (1.01-1.30) under a dominant genetic model for overall CRC. Significant statistical difference was also noted in Asians rather than Caucasians based on the ethnicity subgroups. These results suggested that there is a certain association between rs11615 and the susceptibility of colorectal cancer in the Asian populations.

## 1. Introduction

Colorectal cancer (CRC) is a malignant tumor of the colorectal mucosa epithelial tissue transformed. It is transformed under the factors of genes, diets, environment, and other pathogenic reasons [1]. According to the GLOBOCAN 2016 database, colorectal cancer (CRC) was the third most common cancer accounting for 8% of death among all sites of cancers in the United States [2]. Recurrence and metastasis are the most important causes of death. In the past 20 years, the death rate of CRC decreased continuously in America. However, we cannot ignore a large number of deaths [2]. What is more, CRC morbidity and mortality in China is on the rise in recent years [3]. Currently, CRC has been one of the most threatening tumors affecting people's health worldwide. Many studies have confirmed that not only are dietary habits, environmental factors, and chronic inflammation of the intestinal tract primary elements of colorectal cancer, but the pathogenesis is also influenced by genetic control. Accumulation of DNA damages can cause genomic instability and mutations. Fortunately, 4 major pathways can remove or repair DNA damage, including nucleotide excision repair (NER), mismatch repair (MMR), base excision repair (BER), and double-strand break repair [4]. Repair of DNA was verified to be critical in protecting from cancer-causing agents initially in xeroderma pigmentosum (XP), and subsequently in colon cancer [5]. Mutations of NER-related genes have caused a wide range of attention [6]. ERCC1, as one of the most important rate-limiting enzymes in NER, maps to chromosome 19q13.2 ~ 13.3, length 15 kb, composed of 10 exons, encoding a containing 297 ammonia [7]. So far, many studies have shown that mutations of single nucleotide polymorphisms (SNP) of ERCC1 are associated with multiple types of tumors susceptibility and prognosis [8–12]. A common SNP of ERCC1 gene is located at 118 codon of 19007 *T* > *C* (rs11615, Asn118Asn). As one of the most common SNP of ERCC1, rs11615 polymorphism, a base substitution of ancestral allele C to mutation allele T, has been demonstrated that modify the risk for various cancers, for example, non-small-cell lung cancer, glioma and meningioma, esophageal adenocarcinoma, and gynecology tumors like ovarian and cervical cancer [12–17].

In the past decade, extensive researches were done to find the biomarker for screening for colorectal cancer [18]. However, it needs further exploration. What is more, due to the rapid diagnosis of prostate cancer, the overall cancer incidence declined from 2009 to 2012 [2]. Early screening can decrease the mortality and incidence of colorectal cancer. It can also remove precancerous lesions [19]. Early diagnoses of cancer and precancerous prevention are necessary. Some epidemiological studies have explored the relationship between the susceptibility of CRC and ERCC1 rs11615 variant. Nevertheless, evidence was limited, and the result was inconclusive. The study of Yueh et al. told us the risk of colorectal cancer increased 1.86-fold in people carrying TT genotype on the rs11615 site. They consider the genome becomes unstable if the ERCC1 gene is mutated [20]. The level of mRNA and protein reduced subsequently before cancer happened. But Yang et al. discredited these conclusions [21]. In his study, ERCC1 rs2298881 polymorphism rather than rs11615 is associated with an increased risk of colorectal cancer. We wanted to confirm whether ERCC1 rs11615 could serve as a marker for genetic susceptibility to colorectal cancer. If it is, we can use it to identify high-risk individuals. In addition, there was no meta-analysis focused on the diagnosis of colorectal cancer with ERCC1 rs11615 variant. This paper aims to explore the value of ERCC1 rs11615 gene polymorphism in the diagnosis of colorectal cancer by using meta-analysis.

## 2. Materials and Methods

### 2.1. Search Strategy

A search strategy of literature with the following keywords: (“colorectal neoplasms” or “colorectal cancer” or “colon-rectal cancer”), (“Excision repair cross-complementation group 1” or “ERCC1”), and (“polymorphism” or “genotype” or “variant” or “SNP”) were utilized to search in various databases. We searched keywords in PubMed, Embase, Web of Science, and CNKI, CBM in English or Chinese, respectively. Two authors finished the search independently, and the final search was until the date of July 2017. Publications in English or Chinese were checked. We also checked related references to included studies to find out if there are any other potentially eligible essays.

### 2.2. Selection Criteria

We will intake the publication if it satisfied with following conditions: (1) studies that assessed the polymorphism of ERCC1 rs11615 in CRC patients; (2) using a case-control study or cohort study design; (3) patients in case group are diagnosed with cancer, and populations in control group or based populations are unrelated with CRC clearly, without limit of age, gender, and nationality; (4) each group has described the frequency of genotype in detail; (5) showed data of an odd ratio (OR) with corresponding 95% confidence interval(CI); (6) provided details of detection technology of genotype.

Exclusion criteria: (1) the claim of the study did not mention the relationship of ERCC1 rs11615 polymorphism with colorectal cancer; (2) a meta-analysis or system review; (3) diagnosis of patients is not clear; (4) frequency in each genotype or some important data are not extractable.

Two researchers (Zhifeng Qiu and Min Liu) screened all records independently on the basis of inclusions and exclusions and conducted independent data extraction. They asked help from the third person (Wen Liu) if there is a dispute. We discussed to reach at a consensus. If reports are from the same center or cohort study, we will adopt the one which was the most recent one or most participants.

### 2.3. Data Extraction

We extracted the frequency in each genotype from eligible studies. The first author's name, the year of publication, the object of study in different races, the study design, sample quantity of case and control, based populations, the method of genotyping, and sample source are also extracted by the two authors independently.

### 2.4. Statistical Analysis

We made use of odds ratios (ORs) corresponding to a 95% confidence interval (CI) to assess the strength of the link between ERCC1 rs11615 genotype allele T mutation and CRC compared to allele C. Homozygote model (TT vs. CC), dominant model (TT + TC vs. CC), recessive model (TT vs. TC + CC), and allele model (T vs. C) were applied. We recalculated the ORs after stratification of the ethnicity or other factors that may impact the result. The pool ORs was calculated by the *Z* test (*P* < 0.05 was regarded as having a significant difference). To check the heterogeneity of the between-study, we used *Q* test and *I*-square. If *P* value of *Q* test is less than 0.1, and *I*-square is greater than 50%, we selected a random model. Otherwise, we chose a fixed model [22]. Egger's test and funnel plot were applied to evaluate publication bias. We did the sensitivity analysis to evaluate the stability of the results. STATA (version 12.0) software was applied to calculate the values mentioned above and test whether the genotype frequencies are in accordance with the Hardy-Weinberg equilibrium (HWE) in each control group using Pearson's chi-squared test. *P* < 0.05 (two-sided) was regarded as statistically significant.

### 2.5. Medical Image Security Applications

Medical image security is an important issue when digital images and their pertinent patient information are transmitted across public networks. There are ethical and legal obligations for health care providers to preserve the privacy and confidentiality of patient information, which can contain some of the most intimate information conceivable about an individual. Despite the advantages of electronic medical records (EMR), there is a higher chance of disclosure of information to the public compared to other formats such as paper-based records. Three aspects of security arise in relation to dealing with medical images: confidentiality, reliability, and availability.

## 3. Results

### 3.1. Characteristics of Eligible Studies

Six hundred and eighty-nine articles were found after entering key terms. But only 33 articles were chosen to enter the full-text view phase. Finally, 9 case-control studies, including 2,181 clear-diagnosed cases and 2,828 controls, were analyzed after discarding reviews, duplicates, or those fail to meet the inclusion standards. Details for the literature search and screen were presented in Figure 1. Characteristics of eligible studies have summarized in Table 1. Five studies were conducted in Caucasian populations and four in Asian populations [16–19]. Studies have mentioned that the gender and sex were matched between the case and control group [20, 21, 23–26]. Among these studies, sources of controls were healthy people or hospital-based shown in Table 1. In addition, blood samples for genotyping were used in all studies. The genotype of ERCC1 rs11615 polymorphism was determined using three methods. The polymerase chain reaction-restriction fragment length polymorphism (PRC-RFLP) and TaqMan assay were conducted in nearly all the publications. Matrix-assisted laser desorption ionization-time of flight mass spectrometry (MALDI-TOF MS) was also used in the study of Hou et al. [24]. The genotype distributions were in agreement with HWE (*P* > 0.05) among seven studies, but not in the study of Yueh et al. and Moreno et al. (*P* = 0.049 < 0.05) [20, 25].

### 3.2. Meta-Analysis Results

In this merge meta-analysis, all results of the test for association and heterogeneity were displayed in Table 2. It was detected that significant link occurred between T allele variant in ERCC1 rs11615 site and colorectal carcinoma when every study was pooled into the meta-analysis, containing four genetic models (Table 2, Figure 2), an allele model (OR = 1.13, 95% CI = 1.04 − 1.23, *P* = 0.004, Pheterogeneity = 0.51, and *I*^2^ = 0.0%), a dominant model (OR = 1.14, 95% CI = 1.01 − 1.30, *P* = 0.037, Pheterogeneity = 0.82, and *I*^2^ = 0.0%), a recessive model (OR = 1.19, 95% CI = 1.03 − 1.37, *P* = 0.015, Pheterogeneity = 0.28, and *I*^2^ = 18.8%), and a homozygote model (OR = 1.27, 95% CI = 1.07 − 1.51, *P* = 0.006, Pheterogeneity = 0.41, and *I*^2^ = 3.3%). Stratification by ethnicity confirmed that subjects carrying T genotype increase significantly associated with CRC in Asians. This significance was also found in other genetic models (dominant model: OR = 1.19, 95% CI = 1.00 − 1.41, *P* = 0.046, Pheterogeneity = 0.88, and *I*^2^ = 0.00%; recessive model: OR = 1.36, 95% CI = 1.06 − 1.73, *P* = 0.014, Pheterogeneity = 0.24, and *I*^2^ = 28.00%; homozygote model: OR = 1.43, 95% CI = 1.10 − 1.85, *P* = 0.007, Pheterogeneity = 0.31, and *I*^2^ = 16.7%). However, these associations cannot be found in Caucasians, under any contract model. OR = 1.08, 95% CI = 0.97 − 1.21, Pheterogeneity = 0.51, and *I*^2^ = 0% under the allele model; OR = 1.09, 95% CI = 0.90 − 1.32, Pheterogeneity = 0.51, and *I*^2^ = 0% under the dominant model; OR = 1.11, 95% CI = 0.94 − 1.32, Pheterogeneity = 0.4, and *I*^2^ = 0.7% under the recessive model; OR = 1.16, 95% CI = 0.92 − 1.46, Pheterogeneity = 0.51, and *I*^2^ = 0% under the homozygote model. We reanalyzed based on in accordance with HWE. It came out that no significant association between rs11615 polymorphism and colorectal cancer susceptibility.

### 3.3. Publication Bias and Sensitivity Analysis

With the OR-value as the abscissa, the standard deviation of the log (OR) as the ordinate to draw funnel plots. As displayed in Figure 3, roughly symmetrical was found among studies. And then, proceed to Egger's test. The results are *t* = 1.77 and *P* = 0.12 under a dominant model and *t* = 0.76 and *P* = 0.0.473 under an allele model (data not shown). In the Begg's test, *Pr* > ∣*z* | = 0.348 (continuity corrected) under a dominant model, *Pr* > ∣*z* | = 0.754 (continuity corrected) under an allele model. Begg's funnel plots of other genetic models were shown in Figure 3. In summary, publication bias in this meta-analysis is low. Sensitivity analyses told us that there is no single study that obviously influenced the main result of the summary OR (shown in Figure 4).

## 4. Discussion

The incidence of colorectal cancer between the ages of 30-50 was 50/105 yearly. And the number was double in the age of 50-70. Gradually it rose four times at ages > 70 years [27]. Currently, CRC has been one of the most threatening tumors affecting people's health worldwide. Depending on statistics in America, the mortality of colorectal cancer has markedly dropped owing to carrying out asymptomatic census vigorously. Indeed, it is a matter of utmost urgency to improve the early diagnosis level of colorectal carcinoma in young people to improve the prognosis of patients.

Nucleotide excision repair is a momentous pathway to repair damnifications no matter brought about by endogenic or exogenous reasons. ERCC1-XPF is not similar to other proteins. As a specific endonuclease, it cuts 5′ of the damaged segment in NER. It is also to the recombination and repair of DNA interstrand cross-links [28]. The results of phenotype lead to more serious mutations of ERCC1or XPF than the absence of NER [29]. When the ERCC-XPF is mutated, the capacity of DNA repair decreases and leads to a susceptibility to various decreases such as diverse cancers, genetic disorders Xeroderma pigmentosum (XP), Fanconi anemia (FA), and so on [30–33]. In 2011, Borgesius et al. have used a mouse model mutated with ERCC1 gene to approve that defects of ERCC1 impel acceleration of cognitive decline too [34].

This meta-analysis is an attempt to analyze the potential correlation between the genetic variant of ERCC1 rs11615 and colorectal cancer as well. In this merged analysis, we demonstrated that the susceptible risk of colorectal cancer was associated with the TT variant of ERCC1 Asn118Asn (rs11615) and TC heterozygote compared to wild-type CC homozygote in the overall population. It is the same as Gil et al.'s observation that interaction existed between genotypes of T allele mutant site and morbidity of CRC [35]. However, Skjelbred et al. found that there was no association between the rs11615 polymorphism with the risk of CRC [36]. Gil et al. demonstrated that no evidence for a relationship between ERCC1 rs11615 variant and susceptibility of CRC as well. We have identified that studies of eastern countries contributed to the heterogeneity. We reanalyze by race, and the results showed that the rs11615 polymorphic loci were different for different races. Subgroup analyses of race point out that the correlation between the allele model and the dominant, recessive, homozygote genetic model of ERCC1 rs11615 gene polymorphism and the risk of CRC was statistically significant in Asians, but not in Caucasians. This is similar to the study of meta-analysis by Xie et al. which also pointed out a significant association between 19007 *T* > *C* polymorphism and risk of lung cancer in Asians rather than Caucasians [37]. To note, it occurred differently between subgroups of Asians and Caucasians based on a study by Ding et al. of ERCC1 rs11615 and the risk of head and neck carcinomas as well [38]. We agreed to the suggestion that genetic backgrounds play their part. Some particular environmental exposures, habits, and customs modified the difference among diverse races [37]. Most of the single nucleotide polymorphisms are associated with other genetic polymorphisms and the environment. They regulate the genetic susceptibility of human disease, increase the likelihood of cancer occurrence, and accelerate malignant progression. Interestingly, these associations loss in brain tumors [39]. Li et al. have expounded that no evidence supported the association between cancer and ERCC1 rs11615 in 2007 [40]. To our regret, his study only conducted two articles on colorectal cancer and did not analyze CRC alone. ERCC1 rs11615 mutation has different correlations in different parts of the tumor, and there is a certain degree of disagreement even in the same tumor. Subgroup analyses of HWE and source of control indicated that heterogeneity was from the subgroup of HWE less than 0.05 and population-based studies. The outcomes of publication bias and sensitivity analysis have supported the reliability of this meta-analysis. Since 1990s, it was proved that repair of DNA damage may be suppressed in the case of high expression of ERCC1. This resulted in increased resistance of patients with platinum chemotherapeutic agents [41, 42]. Seetharam et al. got the same conclusion when they used siRNA to silence the ERCC1 in CRC cells and found that CRC cells are sensitive to oxaliplatin-induced apoptosis while ERCC1 gene was inhibited [43]. Expression levels of ERCC1 were an independent factor of overall survival in stage III and IV CRC patients receiving oxaliplatin-based chemotherapy [44, 45]. ERCC1 gene polymorphism is not only associated with tumor susceptibility but also with the efficacy of platinum drugs' treatment in various tumors. Therefore, a combined analysis of ERCC1 and other predictors or prognostic factors is expected to guide the individual clinical diagnosis and treatment.

## 5. Conclusion

Among the nine studies we included, some limitations were discovered when we conducted this meta-analysis. First of all, the source of the case, such as classification of pathological diagnosis, and specific location of cancer was not entirely consistent or not mentioned. We need more messages like family history, exposure history of smoke and alcohol, age, and gender to obtain the adjusted OR. Moreover, detection techniques of disease and diagnostic criteria may also contribute a certain impact to these effects. Although we have collected all the relevant literature as far as possible, we may ignore some of the “gray literatures” such as conference articles, special reports, and so on. What is more, it may result in missing some published literature in other languages. Besides, this study only focused on the SNP loci on the ERCC1 rs11615, without considering other sites caused by the linkage disequilibrium, and further haplotype analysis was not taken into account. The factors given above may cause bias.

With those limitations in mind, our meta-analysis results indicated that ERCC1 rs11615 polymorphism carrying T variant had an association with colorectal cancer in Asians and are still credible. There is evidence to support a certain predictive effect of ERCC1 and tumor susceptibility. In the future, we need more well-designed and large sample size investigations to confirm the precise correlation between ERCC1 rs11615 polymorphism and CRC susceptibility.

## Figures and Tables

**Figure 1:** Flow diagram for screening of articles in this meta-analysis.

**Figure 2:** Forest plots of CRC risk associated with ERCC1 rs11615 under different models stratification by ethnicity. (a) Allele model (T vs. C). (b) Dominant model (TT + TC vs. CC). (c) Recessive model (TT vs. TC + CC). (d) Homozygote model (TT vs. CC).

**Figure 3:** Begg's funnel plots of the association between ERCC1 rs11615 genetic polymorphism and CRC risk under different models. (a) Allele model (T vs. C). (b) Dominant model (TT + TC vs. CC). (c) Recessive model (TT vs. TC + CC). (d) Homozygote model (TT vs. CC).

**Figure 4:** Sensitivity analyses of the summary odds ratio coefficients on the relationships of ERCC1 rs11615 genetic polymorphisms.

**Table 1:** Characteristics of nine eligible studies.

First author	Year	Ethnicity	Country	Case				Control				Total	Genotyping	HWE	Source of control
				CC1	CT1	TT1	Total	CC0	CT0	TT0	Total				
Hansen	2008	Caucasians	DANISH	61	166	168	395	113	349	333	795	1190	PRC-RFLP	0.165	PB
Hou	2014	Asians	CHINA	73	94	37	204	85	90	29	204	408	PRC-RFLP and MALDI-TOF MS	0.514	HB
Ni	2014	Asians	CHINA	117	82	14	213	135	86	19	240	453	TaqMan	0.315	HB
Skjelbred	2006	Caucasians	NORWAY	21	64	68	153	66	185	140	391	544	PRC-RFLP	0.714	PB
Yang	2015	Asians	CHINA	108	121	50	279	134	133	49	316	595	PRC-RFLP	0.100	HB
Yueh	2017	Asians	CHINA	160	131	71	362	180	139	43	362	724	TaqMan	0.049	HB
Gomez	2015	Caucasians	MEXICO	46	47	15	108	58	50	11	119	227	TaqMan	0.962	HB
Moreno	2006	Caucasians	SPAIN	132	138	64	334	123	126	52	301	635	PRC-RFLP	0.049	HB
Gil	2012	Caucasians	POLISH	13	78	42	133	16	48	36	100	233	PRC-RFLP	1.000	HB

PB: Population-based. HB: Hospital-based.

**Table 2:** Summary of ORs (95% CI) with heterogeneity test for ERCC1 rs11615 polymorphism and CRC cancer risk under several genetic models.

Subgroup	No. of studies	T vs. C	*I* ^2^	TT + TC vs. CC	*I* ^2^	TT vs. TC + CC	I^2^	TT vs. CC	*I* ^2^
		OR (95% CI)		OR (95% CI)		OR (95% CI)		OR (95% CI)	
Racial descent									
Asian	4	1.19 (1.05-1.35)^b^	0	1.19 (1.00-1.41)^b^	0	1.36 (1.06-1.73)^b^	28	1.43 (1.10-1.85)^b^	16.7
Caucasian	5	1.08 (0.97-1.21)	0	1.09 (0.90-1.32)	0	1.11 (0.94-1.32)	0.7	1.16 (0.92-1.46)	0
Source of control									
Population-based	2	1.10 (0.85-1.42)	60^a^	1.01 (0.76-1.34)	11.6	1.17 (0.85-1.62)	52.4^a^	1.14 (0.71-1.82)	50.7^a^
Hospital-based	7	1.16 (1.05-1.29)^b^	0	1.18 (1.03-1.36)^b^	0	1.24 (1.03-1.50)^b^	18.5	1.37 (1.12-1.70)^b^	0
HWE									
<0.05	2	1.20 (0.96-1.50)	50.1^a^	1.16 (0.93-1.44)	0	1.43 (0.91-2.26)	60.3^a^	1.46 (0.91-2.35)	57.1^a^
≥ 7.1	7	1.10 (1.00-1.22)	0	1.14 (0.97-1.33)	0	1.12 (0.96-1.32)	0	1.19 (0.97-1.47)	0
Overall	9	1.13 (1.04-1.23)^b^	0	1.14 (1.01-1.30)^b^	0	1.19 (1.03-1.37)^b^	18.8	1.27 (1.07-1.51)^b^	3.3

^a^: Random effect estimate. ^b^: Significant results, *P* < 0.05.

## Data Availability

The datasets used and/or analyzed during the current study are available from the corresponding author on reasonable request.

## References

[1] Pellegrini M. L., Argibay P., Gómez D. E. (2011). Genetics and epigenetics of colorectal cancer. *Acta Gastroenterologica Latinoamericana*.

[2] Rebecca L. (2016). Cancer statistics, 2016. *CA: a Cancer Journal for Clinicians*.

[3] Chen W., Zheng R., Baade P. D. (2016). Cancer statistics in China, 2015. *CA: a Cancer Journal for Clinicians*.

[4] Bao Y., Jiang L., Zhou J. Y. (2013). XRCC1 gene polymorphisms and the risk of differentiated thyroid carcinoma (DTC): a meta-analysis of case-control studies. *PLoS One*.

[5] Shen M. R., Jones I. M., Mohrenweiser H. (1998). Nonconservative amino acid substitution variants exist at polymorphic frequency in DNA repair genes in healthy humans. *Cancer Research*.

[6] Cleaver J. E., Lam E. T., Revet I. (2009). Disorders of nucleotide excision repair: the genetic and molecular basis of heterogeneity. *Nature Reviews Genetics*.

[7] van Duin M., Koken M. H., van den Tol J. (1987). Genomic characterization of the human DNA excision repair gene ERCC-1. *Nucleic Acids Research*.

[8] Arora S., Heyza J., Zhang H. (2016). Identification of small molecule inhibitors of ERCC1-XPF that inhibit DNA repair and potentiate cisplatin efficacy in cancer cells. *Oncotarget*.

[9] Adel Fahmideh M., Schwartzbaum J., Frumento P., Feychting M. (2014). Association between DNA repair gene polymorphisms and risk of glioma: a systematic review and meta-analysis. *Neuro-Oncology*.

[10] Ma Y.-J., Feng S.-C., Hu S.-L., Zhuang S.-H., Fu G.-H. (2014). Association of Rs11615 (C>T) in the excision repair cross-complementing group 1 gene with ovarian but not gynecological cancer susceptibility: a meta-analysis. *Asian Pacific Journal of Cancer Prevention : APJCP*.

[11] Ahmed F. E. (2005). Molecular markers that predict response to colon cancer therapy. *Expert Review of Molecular Diagnostics*.

[12] Zhu J., Hua R.-X., Jiang J. (2014). Association studies of ERCC1 polymorphisms with lung cancer susceptibility: a systematic review and meta-analysis. *PLoS One*.

[13] Zienolddiny S., Campa D., Lind H. (2006). Polymorphisms of DNA repair genes and risk of non-small cell lung cancer. *Carcinogenesis*.

[14] He S.-Y., Xu L., Niu G., Ke P.-Q., Feng M.-M., Shen H.-W. (2012). Predictive value of excision repair cross-complementing rodent repair deficiency complementation group 1 and ovarian cancer risk. *Asian Pacific Journal of Cancer Prevention : APJCP*.

[15] Han S.-S., Kim J. W., Lee S. H. (2012). ERCC1 C19007T polymorphism and the risk and invasiveness of cervical cancer in Korean women. *Asia-Pacific Journal of Clinical Oncology*.

[16] Doecke J., Zhao Z. Z., Pandeya N. (2008). Polymorphisms in MGMT and DNA repair genes and the risk of esophageal adenocarcinoma. *International Journal of Cancer*.

[17] Luo K.-Q., Mu S.-Q., Wu Z.-X., Shi Y.-N., Peng J.-C. (2013). Polymorphisms in DNA repair genes and risk of glioma and meningioma. *Asian Pacific Journal of Cancer Prevention : APJCP*.

[18] Danese E., Montagnana M. (2017). Epigenetics of colorectal cancer: emerging circulating diagnostic and prognostic biomarkers. *Annals of Translational Medicine*.

[19] Bhurgri H., Samiullah S. (2017). Colon cancer screening- is it time yet?. *Journal of the College of Physicians and Surgeons–Pakistan*.

[20] Yueh T.-C., Chou A.-K., Gong C.-L. (2017). The contribution of excision repair cross-complementing group 1 genotypes to colorectal cancer susceptibility in Taiwan. *Anticancer Research*.

[21] Yang H., Li G., Li W. F. (2015). Association between ERCC1 and XPF polymorphisms and risk of colorectal cancer. *Genetics and molecular research : GMR*.

[22] Wang B., Wang D., Huang G., Zhang C., Xu D. H., Zhou W. (2010). XRCC1 polymorphisms and risk of colorectal cancer: a meta-analysis. *International Journal of Colorectal Disease*.

[23] Hansen R. D., Sorensen M., Tjonneland A. (2008). A haplotype of polymorphisms in ASE-1, RAI and ERCC1 and the effects of tobacco smoking and alcohol consumption on risk of colorectal cancer: a Danish prospective case-cohort study. *BMC Cancer*.

[24] Hou R., Liu Y., Feng Y. (2014). Association of single nucleotide polymorphisms of ERCC1 and XPF with colorectal cancer risk and interaction with tobacco use. *Gene*.

[25] Moreno V., Gemignani F., Landi S. (2006). Polymorphisms in genes of nucleotide and base excision repair: risk and prognosis of colorectal cancer. *Clinical Cancer Research*.

[26] Ni M., W-z Z., J-r Q. (2014). Association of ERCC1 and ERCC2 polymorphisms with colorectal cancer risk in a Chinese population. *Scientific Reports*.

[27] De Rosa M., Rega D., Costabile V. (2016). The biological complexity of colorectal cancer: insights into biomarkers for early detection and personalized care. *Therapeutic Advances in Gastroenterology*.

[28] Chipchase M. D., O'Neill M., Melton D. W. (2003). Characterization of premature liver polyploidy in DNA repair (Ercc1)-deficient mice. *Hepatology*.

[29] Ahmad A., Robinson A. R., Duensing A. (2008). ERCC1-XPF endonuclease facilitates DNA double-strand break repair. *Molecular and Cellular Biology*.

[30] Gregg S. Q., Robinson A. R., Niedernhofer L. J. (2011). Physiological consequences of defects in ERCC1-XPF DNA repair endonuclease. *DNA Repair*.

[31] Ahmad A., Enzlin J. H., Bhagwat N. R. (2010). Mislocalization of XPF-ERCC1 nuclease contributes to reduced DNA repair in XP-F patients. *PLoS Genetics*.

[32] Douwel D. K., Hoogenboom W. S., Boonen R. A., Knipscheer P. (2017). Recruitment and positioning determine the specific role of the XPF-ERCC1 endonuclease in interstrand crosslink repair. *The EMBO Journal*.

[33] Bhagwat N., Olsen A. L., Wang A. T. (2009). XPF-ERCC1 participates in the Fanconi anemia pathway of cross-link repair. *Molecular and Cellular Biology*.

[34] Borgesius N. Z., de Waard M. C., van der Pluijm I. (2011). Accelerated age-related cognitive decline and neurodegeneration, caused by deficient DNA repair. *The Journal of Neuroscience*.

[35] Gil J., Ramsey D., Stembalska A. (2012). The C/a polymorphism in intron 11 of the XPC gene plays a crucial role in the modulation of an individual's susceptibility to sporadic colorectal cancer. *Molecular Biology Reports*.

[36] Skjelbred C. F., Saebo M., Nexo B. A. (2006). Effects of polymorphisms in ERCC1, ASE-1 and RAI on the risk of colorectal carcinomas and adenomas: a case control study. *BMC Cancer*.

[37] Xie F., Sun Q., Wu S., Xie X., Liu Z. (2014). Nucleotide excision repair gene ERCC119007T>Cpolymorphism contributes to lung cancer susceptibility: a meta-analysis. *Genetic Testing and Molecular Biomarkers*.

[38] Ding Y. W., Gao X., Ye D. X., Liu W., Wu L., Sun H. Y. (2015). Association of ERCC1 polymorphisms (rs3212986 and rs11615) with the risk of head and neck carcinomas based on case-control studies. *Clinical & Translational Oncology*.

[39] Geng P., Ou J., Li J. (2016). A comprehensive analysis of influence ERCC polymorphisms confer on the development of brain tumors. *Molecular Neurobiology*.

[40] Li Y., Gu S., Wu Q. (2007). No association of ERCC1 C8092A and T19007C polymorphisms to cancer risk: a meta-analysis. *European Journal of Human Genetics*.

[41] Bramson J., Panasci L. C. (1993). Effect of ERCC-1 overexpression on sensitivity of Chinese hamster ovary cells to DNA damaging agents. *Cancer Research*.

[42] Zhen W., Link C. J., O'Connor P. M. (1992). Increased gene-specific repair of cisplatin interstrand cross-links in cisplatin-resistant human ovarian cancer cell lines. *Molecular and Cellular Biology*.

[43] Seetharam R. N., Sood A., Basu-Mallick A., Augenlicht L. H., Mariadason J. M., Goel S. (2010). Oxaliplatin resistance induced by ERCC1 up-regulation is abrogated by siRNA-mediated gene silencing in human colorectal cancer cells. *Anticancer Research*.

[44] Kassem A. B., Salem S. E., Abdelrahim M. E. (2017). ERCC1 and ERCC2 as predictive biomarkers to oxaliplatin-based chemotherapy in colorectal cancer patients from Egypt. *Experimental and Molecular Pathology*.

[45] Mettu N. B., Hurwitz H., Hsu D. S. (2013). Use of molecular biomarkers to inform adjuvant therapy for colon cancer. *Oncology*.

